# Passive Fetal Movement Recognition Approaches Using Hyperparameter Tuned LightGBM Model and Bayesian Optimization

**DOI:** 10.1155/2021/6252362

**Published:** 2021-12-09

**Authors:** Sensong Liang, Jiansheng Peng, Yong Xu, Hemin Ye

**Affiliations:** ^1^College of Electronic Engineering, Guangxi Normal University, Guilin 541004, China; ^2^College of Artificial Intelligence and Manufacture, Hechi University, Hechi 546300, China

## Abstract

Fetal movement is an important clinical indicator to assess fetus growth and development status in the uterus. In recent years, a noninvasive intelligent sensing fetal movement detection system that can monitor high-risk pregnancies at home has received a lot of attention in the field of wearable health monitoring. However, recovering fetal movement signals from a continuous low-amplitude background that is heavily contaminated with noise and recognizing real fetal movements is a challenging task. In this paper, fetal movement can be efficiently recognized by combining the strength of Kalman filtering, time and frequency domain and wavelet domain feature extraction, and hyperparameter tuned Light Gradient Boosting Machine (LightGBM) model. Firstly, the Kalman filtering (KF) algorithm is used to recover the fetal movement signal in a continuous low-amplitude background contaminated by noise. Secondly, the time domain, frequency domain, and wavelet domain (TFWD) features of the preprocessed fetal movement signal are extracted. Finally, the Bayesian Optimization algorithm (BOA) is used to optimize the LightGBM model to obtain the optimal hyperparameters. Through this, the accurate prediction and recognition of fetal movement are successfully achieved. In the performance analysis of the Zenodo fetal movement dataset, the proposed KF + TFWD + BOA-LGBM approach's recognition accuracy and F1-Score reached 94.06% and 96.85%, respectively. Compared with 8 existing advanced methods for fetal movement signal recognition, the proposed method has better accuracy and robustness, indicating its potential medical application in wearable smart sensing systems for fetal prenatal health monitoring.

## 1. Introduction

All over the world, significant public health resources have been devoted to prenatal health surveillance of high-risk mothers with the aim of decreasing perinatal mortality. Despite this, there are 2.6 million stillbirths worldwide each year [1], most of which occur in low- and middle-income countries with relatively poor resources [2, 3]. Stillbirth is often associated with access to appropriate care during pregnancy and delivery [4], and establishing prenatal monitoring can be helpful in decreasing stillbirth [5]. Fetal movement is widely regarded as an important physiological indicator to assess the health of the fetus [6–9]. Fetal movement is defined as any irregular kicking, fluttering, swinging, or rolling and is usually first perceived by the mother at 18 to 20 weeks of pregnancy [10]. The frequency of fetal movements reaches a plateau at 32 weeks of gestation and remains at this level until birth [11, 12]. There is evidence that too little or too much fetal movement in the uterus during the perinatal period can lead to stillbirth [4]. Continuous quantitative recording of fetal movements allows reliable recognition of fetal impairment and enables timely intervention to reduce mortality [5]. Maternal perception of altered or decreased fetal movement is associated with stillbirth [13, 14] and with other adverse outcomes, including maternal-fetal hemorrhage, growth restriction, congenital anomalies, and long-term neurodevelopmental disorders [15–20]. Usually, maternal recurrent perception of fetal movements is considered a sign of fetal health [17, 21, 22]. It is established that maternal perception of fetal movement varies between women [23–25]. Maternal perception of fetal movement is affected by psychological factors and the duration of fetal movement [26]. On the other hand, ultrasound imaging technology, the gold standard for fetal movement detection [32, 49], can provide better reference information. However, this is a long-term electrocardiographic monitoring synchronization process that requires the involvement of highly qualified medical personnel [27]. In addition, this technique cannot be used for a long time for practical and safety reasons [28] and the interference of the ultrasound transducer may distort the Doppler signal.

In recent years, with the rapid development of intelligent sensing devices and the advancement of modern digital information processing technology, automatic recognition of fetal movements using microacceleration sensors and efficient signal processing algorithms has received wide attention [29–42]. The accelerometer sensor is embedded in a wearable device and worn on the abdomen of pregnant women to detect a series of micromovements on the surface of the abdomen. Compared with ultrasound instruments, wearable smart sensing devices have the strength of low monetary cost, easy operation, and long-term fetal movement monitoring at home [41].

*Literature Review of Automatic Fetal Movement Recognition Based on Acceleration Recording Data*. Mesbah et al. [29] designed an accelerometer-based fetal movement detector and proposed a root mean square (RMS) detection method. The use of accelerometers to detect fetal movement signals proved to be more effective than maternal perception and self-counting of fetal movements. However, the RMS method based on amplitude threshold is highly sensitive to noise interference and may not achieve the desired recognition performance. Ryo et al. [30] used a new capacitive accelerometer to record fetal movements during a pregnant woman's nighttime sleep. The recorder holds the promise of accurate and long-term fetal movement health monitoring at home. Layeghy et al. [31] proposed a time-frequency method to analyze the fetal movement signal recorded by acceleration. This method first uses a band-pass filter (BPF) algorithm with bandwidth of 0.5 Hz–45 Hz to denoise the fetal movement signal recorded by acceleration and extract the time-frequency domain (TFD) features of preprocessed signal, and then Support Vector Machine (SVM) model was used for fetal movement recognition (BPF + TFD + SVM). The method gets a good accuracy and sensitivity for the classification of fetal movements. However, the SVM single classifier solves the support vector with the help of quadratic programming, which is difficult to implement for large-scale training samples. Boashash et al. [32] used time-frequency matching pursuit (TFMP) and time-frequency matching filter (TFMF) methods to detect fetal movement signals recorded by accelerometers. The two proposed time-frequency detection methods have low computational complexity and can meet the computing space requirements of most existing microprocessor systems with excellent recognition accuracy. However, it is difficult to build a complete dictionary of fetal movement by empirical observation and does not achieve the desired performance. Altini et al. [33] used a digital band-pass filter with a bandwidth of 1 Hz–20 Hz to denoise the fetal movement signals from the abdominal surface of pregnant women acquired by multiple accelerometers and extract the preprocessed time domain features (TD), and then Random Forest (RF) model was used for fetal movement detection (BPF + TD + RF). The method weighs the relationship between the number of sensors and placement positioning and uses cross validation to achieve realistic and reliable results. kamata et al. [34] used an accelerometer to recognize the number of fetal hiccups in early and late pregnancy. Ryo et al. [35] designed a new accelerometer to record the number of gross fetal movements to determine a normal reference value for such movements. Abeywardhana et al. [36] used time domain (TD) analysis to isolate fetal movements from the raw signals recorded by accelerometers. Zhao et al. [37] used an infinite impulse response (IIR) digital band-pass filter (BPF) algorithm with a bandwidth of 0.5 Hz–20 Hz to denoise the fetal movement signals acquired by accelerometers, and the features after discrete wavelet transform (DWT) were extracted, and then the Fuzzy Adaptive Resonance Theory Mapping (Fuzzy ARTMAP) model was used for fetal movement recognition (BPF + DWT + Fuzzy ARTMAP). The method combines signal preprocessing, threshold detection, and lightweight machine learning algorithms to decrease the computational complexity of the system while maintaining high classification accuracy. However, traditional digital band-pass filters have difficulty in filtering out spectrally mixed fetal movement signals and maternal artifact signals, resulting in a high level of recognition of false positives. Wasalaarachchi et al. [38] proposed an automatic fetal movement counting algorithm based on nonnegative matrix factorization (NMF) and spectral clustering, combined with a home-based wearable device. Delay et al. [39, 47] developed a noninvasive fetal movement recognition system incorporating a convolutional neural network (CNN) hybrid algorithm. Morita et al. [40] used accelerometers to count fetal movements in small for gestational age (SGA) infants and determined that SGA was associated with decreased fetal movements. Zhao et al. [41] used time domain and discrete wavelet domain (TWD) methods to extract potential fetal movement features. Bobrova et al. [42] used a band-pass filter (BPF) algorithm with a bandwidth of 0.5 Hz–20 Hz for denoising. This method has a good suppression effect on the noise outside the frequency band, but it is difficult to filter out the noise signal that overlaps with the spectrum of the fetal movement signal. Martinek et al. [43] used advanced Empirical Mode Decomposition (EMD), Ensemble Empirical Mode Decomposition (EEMD), and Adaptive Wavelet Transform (AWT) signal processing methods for fetal ECG signal denoising. These modern digital signal processing methods provide maximum suppression of interference under some optimal criterion based on some statistical properties of random signals. Lu et al. [44] used the singular spectrum analysis (SSA) method for fetal heart rate signal denoising. The method maintains the same signal trend as conventional denoising algorithms and does not cause signal distortion and attenuation. Du et al. [45] evaluated the relative position of a wearable fetal movement detection device worn on the abdomen of the pregnant woman. Liu et al. [46] used time and frequency domain (TFD) methods to extract fetal movement signal features acquired by multiple pressure sensors. The existing methods for fetal movement signal feature extraction still have shortcomings and do not consider some features such as spectral entropy which indicate the uncertainty and complexity of the signal, so the ideal recognition performance may not be obtained. Vican et al. [48] used an empirical mode decomposition (EMD) algorithm to denoise the signal and extract time domain (TD) features and then used a machine learning (ML) model to recognize fetal movements (EMD + TD + ML). The method can effectively extract the key feature information by fully considering the noise characteristics of the fetal heartbeat signal. Mesbah et al. [49] used a high-pass filter (HPF) algorithm with a cutoff frequency of 0.8 Hz to denoise the fetal movement signal acquired by the accelerometer, and features after independent component analysis (ICA) and discrete wavelet transform (DWT) were extracted, and then Bagging algorithm with Random Forest as its base classifier was used to recognize fetal movement (HPF + ICA + DWT + RF-Bagging). The method uses advanced signal processing techniques to distinguish between real fetal movement signals and artifact signals. However, when the fetal movement signal contains a large noise component, the Bagging algorithm with Random Forest as its base classifier will be overfitted. ML algorithms include Random Forest (RF) [55], Multilayer Perceptron (MLP) [58], Support Vector Machine (SVM) [59], and Logistic Regression (LR) [60] classification models.

In this study, the strengths of Kalman filtering (KF) algorithm, time and frequency domain and wavelet domain (TFWD) feature extraction methods, and Bayesian Optimization algorithm (BOA) for Light Gradient Boosting Machine (LightGBM) model are combined to recognize and evaluate fetal movements (KF + TFWD + BOA-LGBM). The main contributions of this paper are summarized as follows:

1. A KF + TFWD + BOA-LGBM fetal movement recognition framework is developed to effectively solve the problems of difficult fetal movement signal recovery and low recognition accuracy under the background of continuous low-amplitude noise.
2. The KF algorithm is developed for fetal movement signal preprocessing, which is based on some statistical properties of random signals, under some optimal criterion to maximize the suppression of interference while maximizing the recovery of the fetal movement signal, thus achieving the purpose of optimal filtering and solving the problem of spectral mixing of fetal movement signal and interference signal that cannot be separated from each other.
3. A TFWD feature extraction method is developed to improve the recognition performance of the classification model and effectively solve the feature redundancy problem.
4. A BOA-LGBM classification model is developed to improve the fetal movement recognition accuracy by combining Bayesian Optimization algorithm to optimize the hyperparameters of the ensemble learning LightGBM classifier, solving the problems of model overfitting and high computational complexity and the inability of a single classifier to obtain high recognition performance.
5. Comprehensive experiments are designed and conducted to comprehensively demonstrate the efficiency of the KF + TFWD + BOA-LGBM framework by comparing with 8 existing state-of-the-art fetal movement recognition methods, using accuracy, precision, recall, F1-Score, and AUC-ROC as evaluation metrics.

The rest of the arrangements are as follows in Section 2. We first introduce the overall workflow framework of the proposed fetal movement recognition method and then introduce the experimental dataset, fetal movement signal preprocessing algorithm, a feature extraction method, and Bayesian Optimization of LightGBM for fetal movement recognition, respectively, in Section 3. The proposed optimized hyperparameter algorithm, preprocessing algorithm, a feature extraction method, optimized classification algorithm, and recognition method are analyzed and compared with the existing methods, respectively, in Section 4. A brief conclusion is given at the end.

## 2. Materials and Methods

### 2.1. Proposed Methodology

The overall workflow framework of the proposed fetal movement recognition method is shown in Figure 1. Accurate recognition and evaluation of fetal movement are interpreted by combining the strength of Kalman filtering, time domain and frequency domain and wavelet domain feature extraction, and hyperparameter tuned LightGBM model using Bayesian Optimization. In the proposed model, 10-fold cross-validation is used to estimate fetal movement recognition performance.

### 2.2. Dataset Descriptions

For comparative analysis, the proposed method was applied to a publicly available fetal movement dataset. The dataset used throughout this paper is from the Zenodo fetal movement acceleration dataset [61]. The dataset contains fetal movement signals recorded by accelerometers from 16 different pregnant women. The dataset contains signals from an accelerometer positioned on the abdominal wall of the pregnant woman. The accelerometer was ADXL355 from Analog Devices, Inc., with a sampling frequency of 500 Hz.

### 2.3. Preprocessing Using Kalman Filter

In the preprocessing stage, the original acceleration signal is segmented into 2.56 seconds long epochs and then preprocessed using the Kalman filter (KF). The KF is a minimum variance state estimator and the best linear estimator for Gaussian and non-Gaussian noise [62].

Consider the discrete-time system model, expressed by the following equation:

(1) $$\begin{array}{c} x_{k}=A_{k-1}x_{k-1}+B_{k-1}u_{k-1}+w_{k-1},\\ y_{k}=C_{k}x_{k}+v_{k}, \end{array}$$

where *x*_*k*_ and *x*_*k*−1_ are the states at moments *k* and *k* − 1, respectively, *y*_*k*_ ∈ ℝ^*m*^ is the measurement at moment  *k*, *u*_*k*−1_ ∈ ℝ^*p*^ is the known control input, *A*_*k*_ ∈ ℝ^*n*×*n*^ is the known state transfer matrix at moment *k* − 1, *B*_*k*_ ∈ ℝ^*n*×*p*^ is the known input matrix, *C*_*k*_ ∈ ℝ^*m*×*n*^ is the known measurement matrix, *w*_*k*_ ∈ ℝ^*n*^ is the process noise, and *v*_*k*_ ∈ ℝ^*m*^ is the measurement noise. State *x*_0_ ∈ ℝ^*n*^ with estimated ${\hat{x}}_{0|0}$ and error covariance are initialized as follows:

(2) $$\begin{array}{c} P_{0|0}≜E\left[\left(x_{0}-{\hat{x}}_{0|0}\right){\left(x_{0}-{\hat{x}}_{0|0}\right)}^{T}\right], \end{array}$$

where *E*(·) indicates the expectation operator.

The KF equations are shown as follows:

(3) $$\begin{array}{c} {\hat{x}}_{k|k-1}=A_{k-1}{\hat{x}}_{k-1|k-1}+B_{k-1}u_{k-1},\\ P_{k|k-1}=A_{k-1}P_{k-1|k-1}A_{k-1}^{T}+Q_{k-1},\\ K_{k}=P_{k|k-1}C_{k}^{T}{\left(C_{k}P_{k|k-1}C_{k}^{T}+R_{k}\right)}^{-1},\\ {\hat{x}}_{k|k}={\hat{x}}_{k|k-1}+K_{k}\left(y_{k}-C_{k}{\hat{x}}_{k|k-1}\right),\\ P_{k|k}=P_{k|k-1}-P_{k|k-1}C_{k}^{T}{\left(C_{k}P_{k|k-1}C_{k}^{T}+R_{k}\right)}^{-1}C_{k}P_{k|k-1}=\left(1-K_{k}C_{k}\right)P_{k|k-1}, \end{array}$$

where ${\hat{x}}_{k|k-1}$ denotes the a priori estimate of *x*_*k*_, ${\hat{x}}_{k|k}$ denotes the posterior estimate of *x*_*k*_, *K*_*k*_ denotes the Kalman gain, *P*_*k|k*−1_ indicates the state prediction, and *P*_*k|k*_ denotes the updated covariance matrix. *Q*_*k*−1_ and *R*_*k*_ are the state error covariance matrix and the measurement error covariance matrix, respectively. *B*_*k*_ and *u*_*k*−1_ are normally initialized to zero.

When the noise sequences {*x*_0_, *w*_0_,…, *w*_*k*−1_, *v*_1_,…, *v*_*k*_} are Gaussian, uncorrelated, and white, KF generates a minimum variance error estimate ${\hat{x}}_{k|k}$ of the real state *x*_*k*_ for each time *k* given the measurement *y*_1_, *y*_2_,…, *y*_*k*_. When {*x*_0_, *w*_0_,…, *w*_*k*−1_, *v*_1_,…, *v*_*k*_} are non-Gaussian, KF is also the best performing linear filter. The detailed steps of fetal movement signal preprocessing using Kalman filter are shown in Algorithm 1.

### 2.4. Feature Extractions

In this step, the time domain, frequency domain, and wavelet domain (TFWD) features of the preprocessed signal are extracted for training and testing of the classification model. The detailed explanation of TFED feature extraction is shown in Table 1.

### 2.5. Fetal Movement Recognition Using BOA-LightGBM

In this step, the optimal hyperparameters are selected in LightGBM classification and recognition of fetal movements using Bayesian Optimization algorithm (BOA). Finally, the optimal hyperparameter ensemble obtained is used to construct the LightGBM model for recognition and evaluation of fetal movements.

#### 2.5.1. Bayesian Optimization Based on Hyperparameters

Bayesian Optimization algorithm (BOA) is an efficient global optimization method for solving black box functions with comparatively high expense [63]. The Bayesian Optimization algorithm consists of two core components:

1. A Gaussian process (GP) is a combination of a series of random variables that obey a normal distribution within an exponential set. Given a set of measurements *D*_1:*t*_={(*x*_1_, *y*_1_), (*x*_2_, *y*_2_),…, (*x*_*t*_, *y*_*t*_)}, the predicted mean *μ*_*t*_(*x*) and epistemic uncertainty *σ*_*t*_(*x*) at any point *x* in the input space are modeled simultaneously. Here, *x*_*t*_ is the process input and *y*_*t*_ is the corresponding output at time *t*.
2. An acquisition function finds the most promising parameter for the next simulation based on the predicted mean *μ*_*t*_(*x*) and the epistemic uncertainty *σ*_*t*_(*x*).

A GP is defined by its mean function *m* : *x*⟶ℝ^*m*^ and its covariance function *k* : *x* × *x*⟶ℝ^*m*×*n*^, as shown in the following equation:

(4) $$\begin{array}{c} f\left(x\right)∼GP\left(m\left(x\right),k\left(x,x^{\prime }\right)\right), \end{array}$$

where the covariance function *k*(*x*, *x*′), otherwise known as the “kernel,” is used to represent the “smoothness” of the process. If the distance between two points *x* and *x*′ is closer, then the corresponding process outputs *y* and *y*′ will also be closer, and the experimental results are more promising. The squared exponential function (SEF) is the frequent choice of covariance function type, also called radial basis function (RBF).

(5) $$\begin{array}{c} k\left(x,x^{\prime }\right)=\exp\left(-\frac{1}{2\theta^{2}}\left\|x-x^{\prime 2}\right\|\right), \end{array}$$

where parameter *θ* is the length scale used to indicate that the covariance function correlation decreases as the square of the distance between points. In the experimental parameter configuration, the observation model also includes a term representing normally distributed noise *ε* ~ *𝒩*(0, *σ*_noise_^2^) as follows:

(6) $$\begin{array}{c} y=f\left(x\right)+\varepsilon , \end{array}$$

where GP regression can be used to predict the value of the objective function *f*(·) at time *t* + 1 for any position *x*. The result is shown in the following equation:

(7) $$\begin{array}{c} P\left(f_{t+1}|D_{1:t},x\right)=N\left(u_{t}\left(x\right),\sigma_{t}^{2}\left(x\right)\right),\\ u_{t}\left(x\right)=k^{T}{\left[K+\sigma_{\text{noise}}^{2}I\right]}^{-1}y_{1:t},\\ \delta_{t}\left(x\right)=k\left(x,x\right)-k^{T}{\left[K+\delta_{\text{noise}}^{2}I\right]}^{-1}k,\\ k=\left[k\left(x,x_{1}\right),k\left(x,x_{2}\right),\ldots ,k\left(x,x_{t}\right)\right],\\ K=\left[\begin{array}{ccc} k\left(x_{1},x_{1}\right) & \ldots & k\left(x_{1},x_{t}\right)\\ \vdots & \ddots & \vdots \\ k\left(x_{t},x_{1}\right) & \ldots & k\left(x_{t},x_{t}\right) \end{array}\right]. \end{array}$$

With the help of the GP process model, an acquisition function is built to represent the most promising setup for the next computation.

#### 2.5.2. Light Gradient Boosting Machine (LightGBM)

LightGBM is a new member of the boosting ensemble model, developed by researchers at Microsoft and Peking University [53]. LightGBM is an efficient implementation of Gradient Boosting Decision Tree (GBDT) algorithm [64] by introducing Leaf-wise tree growth strategy with the depth limitation and Gradient-based One-side Sampling (GOSS) and Exclusive Feature Bundling (EFB) techniques.

Suppose that there exist datasets obeying independent and identical distributions of dimension *n*, like {*x*_1_,…, *x*_*n*_}, where each independent *x*_*i*_ denotes a vector of dimension *s* in space *χ*^*s*^. In each gradient iteration sampling, the negative gradient of the loss function with respect to the model output can be indicated as {*g*_1_,…, *g*_*n*_}. The decision tree model is assigned to each leaf node based on the maximum information gain value of the segmented feature weights. For GBDT, the information gain after feature segmentation can be described by the variance, which is defined as follows.

Set *O* denotes the training sample with leaf nodes fixed, and the information gain of split point *d* from feature segmentation with *j* is shown in the following equation:

(8) $$\begin{array}{c} V_{j}\left(d\right)=\frac{1}{n_{0}}\frac{{\left(\sum_{x_{i}\in A_{l}}g_{i}\right)}^{2}}{n_{l}^{j}\left(d\right)}+\frac{1}{n_{0}}\frac{{\left(\sum_{x_{i}\in A_{r}}g_{i}\right)}^{2}}{n_{r}^{j}\left(d\right)}, \end{array}$$

where *x*_*i*_ ∈ *A*_*l*_ indicates *x*_*i*_ ≤ *d* and *x*_*i*_ ∈ *A*_*r*_ indicates *x*_*i*_ > *d*. *n*_0_=∑*I*[*x*_*i*_ ∈ *O*], *n*_*l*_^*j*^(*d*)=∑*I*[*x*_*i*_ ∈ *O* : *x*_*ij*_ ≤ *d*], *n*_*r*_^*j*^(*d*)=∑*I*[*x*_*i*_ ∈ *O* : *x*_*ij*_ > *d*], iterate through each segmentation node to find *d*_*j*_^*∗*^=arg max_*d*_*V*_*j*_(*d*), calculate the maximum information gain value *V*_*j*_(*d*_*j*_^*∗*^) from the feature segmentation, then calculate feature *d*_*j*_^*∗*^ to get the segmentation point *j*^*∗*^, and finally divide the data into left and right subleaf nodes.

To exclude the effect of uneven distribution of some data, GOSS updates the information gain by designing a constant multiplier with a small gradient. GOSS first ranks the data according to their absolute magnitude and selects the top *a* examples. Then a random sampling method is used to select *b* examples among the remaining data. Finally, the small gradient data is multiplied with (1 − *a*)/*b*  when updating the segmentation node information gain, which makes the algorithm focus more on the lack of training samples without changing the original data feature distribution. The information gain is calculated by the following equation:

(9) $$\begin{array}{c} V_{j}\left(d\right)=\frac{1}{n_{0}}\frac{{\left(\sum_{x_{i}\in A_{l}}g_{i}+\left(1-a/b\right)\sum_{x_{i}\in B_{l}}g_{i}\right)}^{2}}{n_{l}^{j}\left(d\right)}+\frac{1}{n_{0}}\frac{{\left(\sum_{x_{i}\in A_{r}}g_{i}+\left(1-a/b\right)\sum_{x_{i}\in B_{r}}g_{i}\right)}^{2}}{n_{r}^{j}\left(d\right)}, \end{array}$$

where *V*_*j*_(*d*) denotes the smaller subset of instances and its information gain is used to calculate the segmentation nodes, which can largely reduce the computational complexity.

In this study, taking the fetal movement feature data as an example, we clearly explain the training process of LightGBM model in Algorithm 2.

The following is an explanation of the process of Algorithm 2. ${\hat{y}}_{i}^{\left(t\right)}$ denotes the prediction result of the *i*-th sample at the *t*-th iteration. *f*_*t*_(*x*_*i*_) is the learning function of the *t*-th classification tree. *L*_(*t*)_ is the loss function used to measure the residual between the prediction ${\hat{y}}_{i}^{\left(t\right)}$ and the target *y*_1_. The stopping condition is the completion of the *M*-th iteration of the training process. In addition, the residual value of a sensible loss function can be utilized instead of *M* as the finish iteration condition. If the training residuals of the model are less than the expected set loss value, the training process will be stopped. Two stop iteration conditions can be swapped with each other.

### 2.6. Performance Metrics

The proposed method is evaluated using Accuracy, Precision, Recall, and F1-Score under a confusion matrix. The receiver operating characteristic (ROC) is also an important evaluation indicator, which compares the visualization curves of the true positive and false positive rates. The AUC is defined as the area under the ROC curve. The AUC is a performance metric that measures the merit of a machine learning model. True positive (TP) means that the true class of the sample is a positive case and the model predicts a positive result. True negative (TN) indicates that the true class of the sample is a negative case and the model predicts a negative result. False positive (FP) means that the true class of the sample is a negative case, but the model predicts it to be a positive case. False negative (FN) indicates that the true class of the sample is a positive case, but the model predicts it to be a negative case.

(10) $$\begin{array}{c} \text{Accuracy}=\frac{\text{TP}+\text{TN}}{\text{TP}+\text{TN}+\text{FP}+\text{FN}},\\ \text{Precision}=\frac{\text{TP}}{\text{TP}+\text{FP}},\\ \text{Recall}=\frac{\text{TP}}{\text{TP}+\text{FN}},\\ F1-\text{Score}=\frac{2\times \text{Precision}\times \text{Recall}}{\text{Precision}+\text{Recall}}. \end{array}$$

## 3. Experimental Results

### 3.1. Results and Analysis

In this study, the simulation performance for evaluating fetal movement recognition is analyzed by combining the strengths of Kalman filtering to recover fetal movement signals in a continuous low-amplitude background contaminated by noise, time-frequency domain and wavelet domain feature extraction, and Bayesian Optimization algorithm (BOA) for LightGBM model. The experiments were conducted on a Windows 10 PC with an Intel Core i7-7700 CPU @ 3.6 GHz and 32 GB of RAM. Simulation experiments of the proposed method are conducted using Python 3.8. We analyzed the evaluation metrics like Accuracy, Precision, Recall, F1-Score, and AUC-ROC. The proposed methods are compared for evaluation metrics in signal preprocessing algorithms, feature extraction algorithms, optimization algorithms, and recognition models, respectively.

In this study, the result of fetal movement recognition is expressed as 0, and the result of nonfetal movement recognition is expressed as 1. The experimental analysis is performed using tenfold cross-validation. Previous studies have shown that tenfold cross-validation is beneficial to avoid model overfitting.

### 3.2. Experimental Results with LightGBM Model

The experimental analysis is performed using tenfold cross-validation. Firstly, the raw fetal movement signal is preprocessed using Kalman filter. Secondly, the time domain, frequency domain, and wavelet domain features of the preprocessed signal are extracted. Finally, the hyperparameter values of the LightGBM model were evaluated using Grid Search algorithm (GSA) [50], Random Search algorithm (RSA) [51] and Bayesian Optimization algorithm (BOA) [52].  Table 2 indicates the optimal hyperparameter values obtained by different optimization algorithms for LightGBM model.

To compare the performances of different optimization models, the Accuracy, Precision, Recall, and F1-Score evaluation metrics under confusion matrix are used.  Figure 2 shows the performance analysis of the Accuracy and F1-Score evaluation metrics of LightGBM model using different optimization algorithms.

To better observe the details of different optimization techniques for tuning LightGBM model hyperparameters, Figure 3 shows the kernel density estimation plots for tuning the hyperparametric sampling of the LightGBM model using Grid Search algorithm, Random Search algorithm, and Bayesian Optimization algorithm. As shown in Figure 3, Bayesian Optimization algorithm tends to concentrate around the hyperparameter values and therefore obtains the lowest loss in cross-validation. This demonstrates the advantage of using the Bayesian Optimization algorithm to tune the LightGBM model hyperparameters by spending less time to evaluate promising hyperparameter values.

Table 3 shows the specific average values. As shown in Figures 2 and 3 and Table 3, the LightGBM model with the Bayesian Optimization algorithm outperforms the Grid Search algorithm and the Random Search algorithm in all evaluation metrics. The Grid Search algorithm finds the best combination of hyperparameters by traversing each intersection in the grid, which has the advantage of being effective and suitable for situations where the entire parameter space needs to be searched and the disadvantage of being very computationally expensive and facing dimensional catastrophe. The Random Search algorithm refers to the random search of hyperparameters with the search strategy: for hyperparameters whose search range is distribution, random sampling is performed according to the given distribution, and, for hyperparameters whose search range is list, sampling is performed with equal probability in the given list. The advantage of Random Search is fast calculation, the disadvantage is easy to miss some important information. The Bayesian Optimization algorithm gradually learns to obtain more feedback from the objective function by making initial hyperparameter tuning attempts. Then, different parts of the initial search space are adjusted and sampled. Bayesian Optimization algorithms are more efficient than Grid Search and Random Search algorithms, while avoiding the impact of random search that can miss important information.

### 3.3. Comparative Analysis of the Proposed Preprocessing Algorithm with Previous Studies

To validate the strength of proposed fetal movement signals preprocessing algorithm, the experimental analysis is performed using tenfold cross-validation. The performance of the proposed Kalman filter (KF) preprocessing algorithm is compared with the band-pass filter (BPF) algorithm with a bandwidth of 0.5 Hz–20 Hz [42], Singular Spectrum Analysis (SSA) algorithm [44], Empirical Mode Decomposition (EMD) algorithm, Ensemble Empirical Mode Decomposition (EEMD) algorithm, and Adaptive Wavelet Transform (AWT) algorithm [43]. The existing BPF, SSA, EMD, EEMD, AWT fetal movement signal preprocessing algorithms, and the proposed KF algorithm combined with time domain, frequency domain, and wavelet domain feature extraction methods and Bayesian-optimized LightGBM model are analyzed for tenfold cross validation.  Table 4 shows the comparative analysis of the proposed preprocessing algorithm with the previously studied algorithms, where the parameter type of the EMD technique is the intrinsic modal function (IMF), the parameter type of the EEMD method is the noise standard deviation (STD) and the intrinsic modal function (IMF), and the parameter type of the AWT technique is the wavelet type (WT) and the thresholding (THR).

As shown in Table 4, the proposed Kalman filter preprocessing algorithm for fetal movement signal is the best in all evaluation metrics compared to the existing band-pass filter with a bandwidth of 0.5 Hz–20 Hz algorithm, SSA algorithm, EMD algorithm, EEMD algorithm, and AWT algorithm.

The accuracy of the proposed Kalman filtering algorithm is improved by 1.15%, 1.64%, 2.59%, 4.87%, and 1.38% compared to band-pass filter with a bandwidth of 0.5 Hz–20 Hz algorithm, SSA algorithm, EMD algorithm, EEMD algorithm, and AWT algorithm, respectively.

The advantage of BPF is that each of the useful frequency components and the desired filtered frequency components occupies a different frequency band, and the interference is filtered out by a suitable frequency selection filter to obtain a pure signal. However, there is a possibility of frequency overlap between the fetal movement signal and the interference signal, and then BPF cannot effectively filter out the interference. EMD has the advantage of being data-driven and adaptive, capable of analyzing nonlinear smooth signals. However, EMD obtains IMF components with modal aliasing. EEMD has slightly improved the decomposition efficiency based on EMD algorithm and achieved better results in the field of one-dimensional random signal denoising effectively. However, the EEMD algorithm has high computational complexity and large computational effort. The SSA algorithm maintains the same signal trend as conventional denoising algorithms and does not cause signal distortion and attenuation. In contrast, the Kalman filtering algorithm can estimate the state of a dynamic system from a series of data in the presence of measurement noise when the measurement variance is known. The Kalman filtering algorithm has the advantages of low computational complexity and small computational effort, which can filter out the random noise of continuous low amplitude in the fetal movement signal and recover and correct the fetal movement signal.

### 3.4. Comparative Analysis of the Proposed Feature Extraction Methods with Previous Studies

To validate the strength of the proposed fetal movement signal feature extraction method, the performances of the proposed fetal movement signal time domain, frequency domain, and wavelet domain (TFWD) feature extraction methods are compared with existing time domain (TD) feature extraction methods [36], time domain and wavelet domain (TWD) feature extraction methods [41], and time domain and frequency domain (TFD) feature extraction methods [46]. The existing TD, TWD, TFD fetal movement signal feature extraction methods and the proposed TFWD method combined with Kalman filter algorithm and Bayesian optimized LightGBM model are analyzed for ten-fold cross-validation.

The experimental analysis is performed using tenfold cross-validation.  Figure 4 displays the comparative analysis of proposed feature extraction method with existing research methods.  Table 5 displays the average of the tenfold cross-validation results for different feature extraction methods.

As shown in Table 5, the accuracy performance analysis of the proposed TFWD feature extraction methods improved by 1.98%, 2.14%, and 1.73% compared to the TD feature extraction method, TWD feature extraction methods, and the TFD feature extraction method, respectively.

To validate the performance strength of the proposed TFWD features extraction method, Figure 5 displays the performance analysis of the curves for feature number selection and accuracy.  Figure 6 displays the learning curve for the number of training samples and score. As shown in Figures 5 and 6, the LightGBM model performs increasingly well as the numbers of features and training samples increase, with no overfitting occurring. The existing TD, TWD, and TFD methods for fetal movement signal feature extraction still have shortcomings and do not consider some features such as spectral entropy which indicate the uncertainty and complexity of the signal, so the ideal recognition performance may not be obtained. In contrast, the TFWD method is more comprehensive in feature extraction and fully considers the key detailed features of fetal movement signals in the time domain, frequency domain, and wavelet domain, which makes the model training and classification performance better.

### 3.5. Comparative Analysis of the Proposed Optimization Model with Previous Studies

In order to validate the strength of proposed optimization model, the experimental analysis was performed using tenfold cross-validation. The performance analysis of the proposed Bayesian Optimization algorithm (BOA) [52] for LightGBM model with the existing Grid Search algorithm (GSA) [50], Random Search algorithm (RSA) [51], and genetic programming algorithm (TPTO Classifier) [54] for optimizing the Random Forest (RF) [55] model and Extreme Gradient Boosting (XGBoost) [56] model, respectively, is carried out [57]. The performances are compared and analyzed by changing the optimization model and combining the strengths of Kalman filtering (KF) algorithm and time domain, frequency domain, and wavelet domain (TFWD) feature extraction with tenfold cross-validation.

Figures 7 and 8 show the Accuracy and F1-Score comparison analysis of the proposed Bayesian Optimization algorithm for LightGBM model with existing different optimization models. Figures 9 and 10 show the ROC and Precision-Recall curve performance analysis of the proposed Bayesian Optimization algorithm for LightGBM model with the existing optimization model, respectively.  Table 6 shows the average values of evaluation metrics for different optimization models.

As shown in Figures 7 and 8, the Accuracy and F1-Score evaluation metrics of the proposed BOA-LGBM model are the best compared to the existing optimization models. As shown in Table 6, the accuracy of proposed BOA-LGBM model is improved by 1.81%, 1.48%, 1.15%, 3.79%, 1.97%, and 1.23% compared to the existing methods like RSA-RF, GSA-RF, TPTO-RF, RSA-XGBoost, GSA-XGBoost, and TPTO-XGBoost, respectively.

RF, XGBoost, and LightGBM all belong to ensemble learning, which aims to improve the generalization ability and robustness of the basic learner by combining the prediction results of multiple base learners. RF has the advantage that training can be highly parallelized and handle very-high-dimensional data, with the disadvantage that it tends to overfit in noisy classification or regression problems. XGBoost improves the loss function of the model and adds a regular term for the model complexity. The advantage is the ability to process high-dimensional data in parallel, which largely reduces the computational effort. However, XGBoost uses presorting, which requires presorting the features of the nodes before iteration and then traversing to select the best segmentation point, and the algorithm is more time-consuming when the data volume is large. In contrast, LightGBM uses histogram algorithm, which occupies low memory and has lower complexity of data segmentation. In addition, LightGBM uses deep optimization and leaf-wise growth strategy, which selects the node with the greatest gain from the current leaf for segmentation each time and iterates cyclically to prevent overfitting.

### 3.6. Comparative Analysis of the Proposed Model with Previous Studies

The KF + TFWD + BOA-LGBM proposed is analyzed and compared with various existing fetal movement signal preprocessing, feature extraction, and recognition methods, namely, band-pass filter with a bandwidth of 0.5 Hz–45 Hz preprocessing and time and frequency domain feature selection and Support Vector Machine classification methods (BPF + TFD + SVM) [31], band-pass filter with a bandwidth of 1 Hz–20 Hz preprocessing and time domain feature extraction and Random Forest classification methods (BPF + TD + RF) [33], band-pass filter with a bandwidth of 0.5 Hz–20 Hz preprocessing and Discrete Wavelet Transform feature extraction and Fuzzy Adaptive Resonance Theory Mapping classification methods (BPF + DWT + Fuzzy ARTMAP) [37], Empirical Mode Decomposition preprocessing and time domain feature extraction and machine learning classification methods (EMD + TD + ML) [48], high-pass filter with a cutoff frequency of 0.8 Hz preprocessing and Independent Component Analysis and Discrete Wavelet Transform feature extraction and Bagging classification methods with Random Forest as its base classifier (HPF + ICA + DWT + RF-Bagging) [49]. ML algorithms include Random Forest (RF) [55], Multilayer Perceptron (MLP) [58], Support Vector Machine (SVM) [59], and Logistic Regression (LR) [60] classification models.

In order to validate the strength of the proposed fetal movement classification model, the experimental analysis is performed using tenfold cross-validation. As shown in Figures 11 and 12, the accuracy and F1-Score evaluation metrics of the proposed KF + TFWD + BOA-LGBM model are compared with existing models. As shown in Figures 13 and 14, the ROC curves and Precision-Recall curves of the proposed KF + TFWD + BOA-LGBM model are compared with the existing models.  Table 7 displays the average values of evaluation metrics for different models with 10-fold cross-validation.

As shown in Table 7, the accuracy of the proposed KF + TFWD + BOA-LGBM model for fetal movement recognition is higher than those of the existing methods such as BPF + TFD + SVM, BPF + TD + RF, BPF + DWT + Fuzzy ARTMAP, EMD + TD + RF, EMD + TD + MLP, EMD + TD + SVM, EMD + TD + LR, and HPF + ICA + DWT + RF-Bagging, improving by 11.38%, 2.14%, 3.47%, 2.06%, 6.85%, 6.93%, 7.1%, and 2.88%, respectively. The F1-Score of proposed KF + TFWD + BOA-LGBM model for fetal movement recognition was higher than those of the existing methods such as BPF + TFD + SVM, BPF + TD + RF, BPF + DWT + Fuzzy ARTMAP, EMD + TD + RF, EMD + TD + MLP, EMD + TD + SVM, EMD + TD + LR, and HPF + ICA + DWT + RF-Bagging, improving by 7.07%, 1.42%, 2.6%, 1.37%, 4.75%, 4.61%, 4.85%, and 2.45%, respectively.

For existing fetal movement signal preprocessing algorithms. BPF has the advantage that each of the fetal movement signal components and the desired filtered frequency components occupies a different frequency band. Then, the interference is filtered out by a suitable frequency selection filter to obtain a pure signal. However, BPF cannot effectively filter out the interference when there is a possibility of spectral overlap between the fetal movement signal and the interfering signal. EMD has the advantage of being data-driven and adaptive, capable of analyzing nonlinear smooth signals. However, EMD obtains IMF components with modal aliasing, which can lead to erroneous time-frequency fetal movement signals. The advantages of ICA allow for blind source separation of fetal movement signals. However, the separation of the fetal movement signal components by the ICA algorithm leads to inconsistency between the amplitude and the source signal. In addition, the algorithm may not be applicable when the assumptions are not satisfied. In contrast, the KF algorithm can estimate the state of a dynamic system from a series of data in the presence of measurement noise when the measurement variance is known. The Kalman filtering algorithm has the advantages of low computational complexity and small computational effort, which can filter out the random noise of continuous low amplitude in the fetal movement signal and recover and correct the fetal movement signal.

For existing fetal movement classification algorithm, the SVM classification algorithm uses kernel functions to map to higher-dimensional spaces and solve nonlinear classification problems. However, the algorithm is difficult to implement for large training samples and is sensitive to the choice of parameters and kernel functions. The MLP algorithm consists of many identical simple processing units combined in parallel, with a high degree of parallelism and good fault tolerance and associative memory. However, the problem of selecting the number of implicit nodes for the network of this algorithm remains a challenge so far, and the learning speed is slow and easy to fall into local limit values. The LR algorithm is computationally inexpensive and can handle large data using fewer resources, but it tends to underfit and has low classification accuracy. Fuzzy ARTMAP belongs to lightweight neural network algorithm, which is computationally inexpensive and has good performance and wide applicability, but the classification process agrees to overfitting. RF has the advantage that training can be highly parallelized and handle very-high-dimensional data, with the disadvantage that it tends to overfit in noisy classification or regression problems. In contrast, LightGBM uses histogram algorithm, which occupies low memory and has lower complexity of data segmentation. In addition, LightGBM uses deep optimization, leaf-wise growth strategy, which selects the node with the greatest gain from the current leaf for segmentation each time and iterates cyclically to prevent overfitting.

## 4. Conclusion

In this paper, the strengths of Kalman filtering, time and frequency domain and wavelet domain, and Bayesian Optimization LightGBM model are combined for the accurate prediction and recognition of fetal movements. Firstly, the Kalman filtering (KF) algorithm is used to recover the fetal movement signal in a continuous low-amplitude background contaminated by noise. Secondly, the time domain, frequency domain, and wavelet domain (TFWD) features of the preprocessed fetal movement signal are extracted. Finally, the Bayesian Optimization algorithm is used to optimize the LightGBM classifier to obtain the optimal hyperparameters. In this manuscript, Kalman filtering combined with time and frequency domain and wavelet domain feature extraction and Bayesian Optimization LightGBM model provides the best recognition results based on prediction and detection. In the performance analysis of the Zenodo fetal movement dataset, the proposed KF + TFWD + BOA-LGBM model has a higher recognition accuracy compared to the existing methods such as BPF + TFD + SVM, BPF + TD + RF, BPF + DWT + Fuzzy ARTMAP, EMD + TD + RF, EMD + TD + MLP, EMD + TD + SVM, EMD + TD + LR and HPF + ICA + DWT + RF-Bagging, improving by 11.38%, 2.14%, 3.47%, 2.06%, 6.85%, 6.93%, 7.1%, and 2.88%, respectively. The experimental results showed that the proposed KF + TFWD + BOA-LGBM model is more robust to predict and recognize fetal movements. The proposed method has significant medical value and broad application prospects for the application of intelligent sensing-based technology to clinical fetal movement detection.

## Figures and Tables

**Figure 1:** Overall workflow framework of the proposed fetal movement recognition method.

**Figure 2:** Performance analyses of the Accuracy and F1-Score evaluation metrics of LightGBM model with tenfold cross-validation using different optimization algorithms.

**Figure 3:** The kernel density estimation plots for tuning the hyperparametric sampling of the LightGBM model using Grid Search algorithm, Random Search algorithm, and Bayesian Optimization algorithm.

**Figure 4:** The comparative analysis of proposed feature extraction method with existing research methods.

**Figure 5:** The performance analysis of the curves for feature number selection and accuracy.

**Figure 6:** The learning curve for the number of training samples and score.

**Figure 7:** The accuracy comparison analysis of the proposed Bayesian Optimization algorithm for LightGBM model with existing different optimization models.

**Figure 8:** F1-Score comparison analysis of the proposed Bayesian Optimization algorithm for LightGBM model with existing different optimization models.

**Figure 9:** The ROC curve performance analysis of the proposed BOA-LGBM model with the existing optimization model.

**Figure 10:** Precision-Recall curve performance analyses of the proposed BOA-LGBM model with the existing optimization model.

**Figure 11:** The accuracy evaluation metrics of the proposed KF + TFWD + BOA-LGBM model are compared with existing models.

**Figure 12:** The F1-Score evaluation metrics of the proposed KF + TFWD + BOA-LGBM model are compared with existing models.

**Figure 13:** ROC curves of proposed KF + TFWD + BOA-LGBM model are compared with the existing models.

**Figure 14:** Precision-Recall curves of proposed KF + TFWD + BOA-LGBM model are compared with the existing models.

**Algorithm 1:** Preprocessing of fetal movement signal using Kalman filter.

**Algorithm 2:** The training process of LightGBM model.

**Table 1:** The detailed explanation of TFWD features extraction.

Feature no.	Feature	Description
1	T_Mean	The time domain signal mean.
2	T_STD	The time domain signals standard deviation.
3	T_ Median	The time domain signals median.
4	T_Max	The time domain signals maximum.
5	T_Min	The time domain signals minimum.
6	T_IQR	The time domain signals interquartile range.
7	T_ Energy	The time domain signals energy.
8	T_WF	The time domain signals waveform factor.
9	T_CF	The time domain signals crest factor.
10	T_PF	The time domain signals pulse factor.
11	T_MF	The time domain signals margin factor.
12	F_FIM	The frequency index of the spectrum maximum.
13	F_SM	Spectrum maximum.
14	F_FISM	The frequency index of the spectrum submaximum.
15	F_SSM	Spectrum submaxima.
16	F_Mean	The mean of the spectrum.
17	F_ Skewness	Spectrum skewness.
18	F_ Kurtosis	Spectrum kurtosis.
19	F_ Entropy	Spectrum entropy.
20	W_ Energy	The sum of energy for each subband signal after wavelet transforms.
21	W_Mean	The sum of mean for each subband signal after wavelet transforms.
22	W_STD	The sum of standard deviations for each subband signal after wavelet transforms.

**Table 2:** Optimal hyperparameter values are obtained by different optimization algorithms for LightGBM model.

Model	Parameters	Grid Search	Random Search	Bayesian Optimization
LightGBM	N_estimators	90	50	51
	Max_depth	8	9	5
	Num_leaves	50	225	63
	Subsample	0.7	0.9	0.8863
	Colsample_bytree	0.7999	0.8899	0.9079
	Min_child_samples	4	7	8

**Table 3:** Performance analysis results of LightGBM model using different optimization algorithms.

Metrics	Grid Search (%)	Random Search (%)	Bayesian Optimization (%)
Accuracy	92.91	93.16	94.06
Precision	94.12	94.09	94.48
Recall	96.29	96.64	97.56
F1-Score	95.12	95.29	95.94
AUC-ROC	96.93	96.6	96.85

**Table 4:** The comparative analysis of the proposed preprocessing algorithm with the previously studied algorithms.

Authors	Method	Accuracy (%)	Precision (%)	Recall (%)	F1-Score (%)	AUC-ROC (%)
Bobrova et al. [42]	BPF (0.5 Hz–20 Hz)	92.91	93.67	96.87	95.16	95.93
Lu et al. [44]	SSA	92.42	92.7	97.21	94.85	94.69
Martinek et al. [43]	EMD (IMF = 3 + 4 + 5)	92.17	92.39	97.21	94.67	94.22
	EMD (IMF = 4)	90.77	90.84	96.98	93.75	94.59
	EEMD (STD = 0.2, IMF = 4)	88.53	90.39	94.08	92.14	91.80
	EEMD (STD = 0.2, IMF = 4 + 5)	89.69	89.93	96.52	93.04	92.83
	EEMD (STD = 0.3, IM = 4)	89.28	91.05	94.31	92.62	93.30
	EEMD (STD = 0.3, IM = 4 + 5)	89.27	90.54	95.12	92.69	93.14
	AWT (WT = db 4, THR = hard)	92.82	93.39	96.98	95.09	96.44
	AWT (WT = db4, THR = soft)	92.83	93.73	96.63	95.08	96.79
	AWT (WT = sym4, THR = hard)	92.58	93.60	96.40	94.90	95.64
	AWT (WT = sym4, THR = soft)	92.49	93.29	96.63	94.85	96.06
Proposed	Kalman filter	94.06	94.48	97.56	95.94	96.85

**Table 5:** The average of the tenfold cross-validation results for different feature extraction methods.

Authors	Method	Accuracy (%)	Precision (%)	Recall (%)	F1-Score (%)	AUC-ROC (%)
Abeywardhana et al. [36]	TD	92.08	93.05	96.29	94.57	96.33
Zhao et al. [41]	TWD	91.92	92.96	96.29	94.49	96.72
Liu et al. [46]	TFD	92.33	93.38	96.29	94.74	96.67
Proposed	TFWD	94.06	94.48	97.56	95.94	96.85

**Table 6:** The average values of evaluation metrics for different optimization models with tenfold cross-validation.

Authors	Method	Accuracy (%)	Precision (%)	Recall (%)	F1-Score (%)	AUC-ROC (%)
Valarmathi et al. [57]	RSA-RF	92.25	93.76	95.71	94.76	96.86
	GSA-RF	92.58	93.77	96.17	94.81	97.03
	TPTO-RF	92.91	93.73	96.40	94.85	96.78
	RSA-XGBoost	90.27	94.69	91.64	93.07	93.73
	GSA-XGBoost	92.09	92.89	96.41	94.56	95.83
	TPTO-XGBoost	92.83	93.46	96.87	95.08	96.33
Proposed	BOA-LGBM	94.06	94.48	97.56	95.94	96.85

**Table 7:** The average values of evaluation metrics for different models with 10-fold cross-validation.

Authors	Method	Accuracy (%)	Precision (%)	Recall (%)	F1-Score (%)	AUC-ROC (%)
Layeghy at el [31]	BPF + TFD + SVM	82.68	82.29	96.75	88.87	87.56
Altini et al. [33]	BPF + TD + RF	91.92	93.25	96.29	94.52	97.19
Zhao et al. [37]	BPF + DWT + Fuzzy ARTMAP	90.59	93.09	93.69	93.34	88.23
Vican et al. [48]	EMD + TD + RF	92.0	92.53	96.29	94.57	96.77
	EMD + TD + MLP	87.21	90.48	91.76	91.19	91.37
	EMD + TD + SVM	87.13	88.96	94.19	91.33	90.45
	EMD + TD + LR	86.96	89.53	93.03	91.09	90.99
Mesbah et al. [49]	HPF + ICA + DWT + RF-Bagging	91.18	93.16	94.43	93.49	94.90
Proposed	KF + TFWD + BOA-LGBM	94.06	94.48	97.56	95.94	96.85

## Data Availability

The data used for this study are available in publicly available datasets, available online at https://doi.org/10.5281/zenodo.3544631.
